# Genetic variability of DNA repair mechanisms influences treatment outcome of gastric cancer

**DOI:** 10.3892/ol.2015.3510

**Published:** 2015-07-17

**Authors:** CHANGMAO DING, HUIYU ZHANG, KUISHENG CHEN, CHUNLIN ZHAO, JIANBO GAO

**Affiliations:** 1 Department of Radiology, The First Affiliated Hospital of Zhengzhou University, Zhengzhou, Henan 450052, P.R. China; 2 Department of Pathology, The First Affiliated Hospital of Zhengzhou University, Zhengzhou, Henan 450052, P.R. China; 3 Department of General Surgery, The First Affiliated Hospital of Zhengzhou University, Zhengzhou, Henan 450052, P.R. China

**Keywords:** single nucleotide polymorphism, DNA repair pathway, gastric cancer, clinical outcome

## Abstract

The aim of the current study was to investigate the role of polymorphisms in DNA repair pathways on the clinical outcome of gastric cancer patients treated with platinum-based chemotherapy. A total of 380 gastric cancer patients treated with platinum-based chemotherapy were included in the present study. The genotypes of *ERCC1* rs11615 (Asn118Asn) and rs3212986 (*197G>T), *ERCC2* rs1799793 (Asn312Asp) and rs13181 (Lys751Gln), *NBN* rs1805794 (Gln185Gln) and rs1063054 (*1209A>C), *RAD51* rs1801321 (−61G>T) and rs12593359 (*502T>G), and *XRCC3* rs861539 (Thr241Met) were determined by polymerase chain reaction-restriction fragment length polymorphism, according to the manufacturer's instructions. The TC+CC genotypes of *ERCC1* rs11615 and GA+AA genotypes of *ERCC2* rs1799793 were found to be associated with improved response to chemotherapy, with an adjusted odds ratio of 1.66 (95% CI, 1.07–2.56) and 1.61 (95% CI, 1.05–2.49), respectively. Based on the results of Cox analysis, patients with TC+CC genotypes of *ERCC1* rs11615 and GA+AA genotypes of *ERCC2* rs1799793 exhibited a significantly decreased risk of mortality, with hazard ratios of 1.71 (95% CI, 1.06–2.72) and 1.97 (95% CI, 1.28–3.03), respectively. In conclusion, these results suggest that *ERCC1* rs11615 and *ERCC2* rs1799793 in the DNA repair pathways may be used as predictive factors of the clinical outcome in gastric cancer patients.

## Introduction

Gastric cancer is the fifth most common malignancy worldwide. It is estimated that 952,000 new gastric cancer cases and 723,000 gastric cancer-associated mortalities occurred in 2012 (1). Over 70% of gastric cancer cases occur in developing countries, with half of these occurring in China (1,2). Surgery is the primary method for treating early-stage disease; however, a high proportion of patients develop local or distant recurrence even after receiving surgical treatment. At present, neoadjuvant chemotherapy followed by surgery is widely used for gastric cancer patients, and this has been demonstrated to improve survival times (3).

Although the outcomes of patients with gastric cancer have been improved significantly by platinum-based chemotherapy, its efficacy and toxicity are highly variable in different patients (4,5). Recent increasing evidence has indicated that hereditary factors are crucial in such individual differences in the response to platinum-based chemotherapy (6–10). Single nucleotide polymorphisms (SNPs) may lead to changes in the activity of enzymes and transporters that are involved in platinum-based drug elimination, and may affect survival and treatment-associated toxicity (11).

Platinum analogs can bind to DNA, forming adducts (intrastrand and interstrand crosslinks) and inhibiting DNA replication (12). DNA repair mechanisms are, therefore, important factors determining the response to chemotherapy. Intrastrand crosslinks represent the majority of chemotherapy-induced DNA damage, and nucleotide excision repair (NER) is the predominant mechanism involved in their repair (13). However, as interstrand crosslinks affect both DNA strands, they are more cytotoxic compared with intrastrand crosslinks, and their repair through homologous recombination repair (HRR) and translesion polymerases is crucial for genomic stability (14–16).

All DNA repair pathways are complex and involve numerous different enzymes. The NER pathway is primarily important in helix-distorting DNA lesions and cytotoxic DNA interstrand crosslinks (17). Two genes encoding enzymes in the NER pathway are frequently associated with resistance to platinum-based chemotherapy: Excision repair cross-complementation group 2 (*ERCC2*) and *ERCC1*.

Other complex DNA damage requires alternative mechanisms, such as HRR, for successful repair. In the HRR pathway, nibrin (NBN) is one of the complexes involved in the recognition of DNA damage, while RAD51 recombinase (RAD51) and X-ray complementing defective repair in Chinese hamster cells 3 (XRCC3) catalyze homologous search and strand invasion.

The aim of the current study was to investigate the role of polymorphisms in DNA repair pathways in the clinical outcome of gastric cancer patients treated with platinum-based chemotherapy.

## Patients and methods

### 

#### Patients

A total of 380 gastric cancer patients treated with platinum-based chemotherapy were enrolled at the First Affiliated Hospital of Zhengzhou University (Zhengzhou, China) between January 2008 and January 2011. All the patients were Han Chinese with newly diagnosed and histopathologically confirmed gastric cancer. None of the patients had previously received systemic anticancer chemotherapy. Bone marrow reserve and normal renal function, liver function and cardiac function prior to chemotherapy were necessary for inclusion in the study. Patients who had severe concomitant systemic disorders and were unable to receive chemotherapy, presented metastasis with symptoms, lacked comprehensive data or developed other diseases (such as neural system diseases) were excluded from the study, as these symptoms or diseases may affect the safety of patients or the evaluation of the results. All patients provided written informed consent for blood sample collection to establish the clinical significance of genetic polymorphisms in the response to platinum-based chemotherapy. The study was approved by the review board of the First Affiliated Hospital of Zhengzhou University.

#### Assessment of treatment outcome

Demographic, clinical and treatment parameters were obtained from the medical records. Tumor response to chemotherapy was evaluated based on the World Health Organization criteria (18). All the patients were followed-up until 30th December 2013, with a median follow-up time of 29.6 months (range, 2–60 months). Patients were followed-up by telephone every four weeks until mortality or the end of the study.

The overall survival (OS) was defined as the period from the beginning of treatment until mortality or the end of the follow-up period. Complete remission and partial remission were considered to be responsive, while stable disease and progressive disease were considered to be non-responsive. Patients without an event or mortality at the time of the analysis were censored at the date of the last follow-up.

Individuals who had smoked ≥1 cigarette per week for more than half a year previously were defined as smokers, whilst individuals who had consumed alcoholic beverages at least once per week for more than half a year previously were defined as drinkers.

#### DNA extraction and genotyping

Genomic DNA was isolated from peripheral blood lymphocytes using a QIAamp DNA Blood Mini kit (Qiagen, Hilden, Germany) according to the manufacturer's instructions. The genotypes of *ERCC1* rs11615 (Asn118Asn) and rs3212986 (*197G>T), *ERCC2* rs1799793 (Asn312Asp) and rs13181 (Lys751Gln), *NBN* rs1805794 (Gln185Gln) and rs1063054 (*1209A>C), *RAD51* rs1801321 (−61G>T) and rs12593359 (*502T>G), and *XRCC3* rs861539 (Thr241Met) were determined by polymerase chain reaction (PCR)-restriction fragment length polymorphism analysis, according to manufacturer's instructions. The PCR reaction was conducted in a 25 µl reaction solution with 25 mM MgCl_2_, 1 ng/µl of each primer and 2 mM deoxynucleotide triphosphates, and 1.25 units of Taq polymerase (Takara Biotechnology Co., Ltd., Dalian, China) as well as 0.5 µl 5X PCR buffer (Takara Biotechnology Co., Ltd.). The cycling program of the PCR reaction conditions commenced with a 95°C denaturation step lasting for 10 min, followed by 40 cycles of 95°C for 30 sec, 62°C for 30 sec and 72°C for 30 sec, and an extension at 72°C for 10 min. A total of ~5% of the samples were repeatedly genotyped, and the results were 100% concordant.

#### Statistical analysis

All statistical analyses were conducted using STATA statistical software version 9.0 (StataCorp LP, College Station, TX, USA). Frequencies were used to describe the distribution of categorical variables, while the median and interquartile range were used for continuous variables. A standard χ^2^ test was used to assess deviation from the Hardy-Weinberg equilibrium. The Cox proportional hazards model was used in the survival analysis to calculate the hazard ratio (HR) and 95% confidence interval (CI). Survival distributions were estimated by using the Kaplan-Meier method. Logistic regression was used to assess the effect of genetic polymorphisms or clinical variables on binary treatment outcomes, and odds ratios (ORs) and their 95% CIs were determined. A dominant genetic model was used in all statistical analyses. All P-values were two-sided, and a P<0.05 was considered to indicate a statistically significant difference.

## Results

### 

#### Patient demographic and clinical characteristics

The demographic and clinical characteristics of the patients are listed in Table I. The ages of the patients were between 23 and 82 years at diagnosis (mean ± standard deviation, 58.7±16.3 years). Among the included 380 gastric cancer patients, 244 (64.21%) patients were men, 136 (35.79%) were women, 166 (43.68%) were smokers, 208 (54.74%) consumed alcohol, 172 (45.26%) had intestinal type gastric cancer, 164 (43.16%) had signet ring type gastric cancer, 248 (65.26%) had a poor histological grade, and 234 (61.58%) were of TNM stage III–IV (19). Using the Cox proportional hazards regression analysis, patients with stage III–IV tumors were found to have a significantly higher risk of mortality associated with gastric cancer compared with those with stage I–II disease, with a HR of 2.54 (95% CI, 1.46–3.28; P=0.007).

#### Association between SNPs and response to chemotherapy

The association between the investigated SNPs and response to chemotherapy in gastric cancer patients are listed in Table II. Among the 380 gastric cancer patients, 223 (58.68%) exhibited a good response to chemotherapy. Following adjustment for clinical variables, the TC+CC genotypes of *ERCC1* rs11615 were correlated with a significantly improved response to chemotherapy compared with that of the reference genotype (TT), with an adjusted OR of 1.66 (95% CI, 1.07–2.56; P=0.02). Furthermore, the GA+AA genotypes of *ERCC2* rs1799793 were associated with a significantly better response to chemotherapy (OR, 1.61; 95% CI, 1.05–2.49) compared with that of the GG genotype (P=0.02).

#### Association between SNPs and survival

The Kaplan-Meier method and Cox regression analysis were conducted to assess the role of the 9 investigated SNPs in the OS of gastric cancer patients (Table III). This analysis revealed that *ERCC1* rs11615 was associated with OS of gastric cancer: Patients with the TC+CC genotypes had a longer survival time compared with those with the common TT genotype (33.20 vs. 23.30 months; log-rank P=0.017). Furthermore, the GA+AA genotypes were associated with a longer survival time compared with that of the GG genotype (34.80 vs. 23.10 months; log-rank P=0.005).

The Cox regression analysis revealed that patients with TC+CC genotypes of *ERCC1* rs11615 exhibited a significantly reduced risk of mortality compared with patients with the TT genotype (HR, 1.71; 95% CI, 1.06–2.7; P=0.02; Fig. 1). For *ERCC2* rs1799793, the GA+AA genotypes were found to be significantly associated with a lower risk of mortality from gastric cancer compared with that of the GG genotype (HR, 1.97; 95% CI, 1.28–3.03; P=0.001; Fig. 2).

## Discussion

In the present study, the effect of SNPs in genes involved in DNA repair mechanisms on the response to treatment and survival in gastric cancer patients treated with platinum-based chemotherapy was investigated. The genotypes of *ERCC1* rs11615 and *ERCC2* rs1799793 were revealed to affect the response to chemotherapy, and were associated with the OS in gastric cancer patients.

Platinum-based chemotherapy is a commonly used chemotherapeutic strategy that exerts a cytotoxic effect primarily through the formation of various types of DNA lesions. DNA repair mechanisms may, therefore, be important in determining the response of tumors to platinum-based chemotherapy (20). NER enzymes are among the most important factors that are able to modify susceptibility to platinum-based chemotherapy; however, other mechanisms involved in the repair of complex forms of DNA damage, including HRR, may also contribute to differences in response between individual patients (21). The current study revealed that *ERCC1* rs11615 is associated with the outcome in cases of gastric cancer treated with chemotherapy. A previous study has also reported that *ERCC1* rs11615 was associated with the response to chemotherapy and clinical outcome in cases of gastric cancer (22). Li *et al* (23) reported that individuals carrying *ERCC1* rs11615 polymorphisms had an increased risk of mortality from gastric cancer compared with the risk of individuals carrying the common genotype, and this genetic polymorphism may contribute substantially to the future design of individualized treatments for gastric cancer patients. Another study has previously investigated the association between three functional SNPs in DNA repair pathways and the clinical outcome of 940 cases of gastric cancer in a Chinese population, and reported that *ERCC1* rs11615 did not affect the OS of gastric cancer patients (23). However, a study by Lu *et al* (24) reported the opposite conclusions. The authors conducted a study including 447 patients in China, and reported that the T allele of *ERCC1* rs11615 decreased the risk of mortality from gastric cancer (19). Such discrepancies among the reports may be explained by differences in the ethnicities of the studied patients, sample size and study design, and also by chance. Further studies are required in order to confirm the association between *ERCC1* rs11615 and clinical outcome in cases of gastric cancer.

The present study also revealed that *ERCC2* rs1799793 is an important factor influencing the response to chemotherapy and OS in cases of gastric cancer, following adjustment for multiple potential risk factors. A previous study reported that the non-synonymous *ERCC2* rs1799793 SNP is associated with a reduced DNA repair capacity compared with that of the common genotype (25). The current results are in concordance with the proposed biological effect of *ERCC2* rs1799793, as a lower repair capacity may lead to increased DNA damage and therefore to greater efficacy of chemotherapy, but also increased toxicity (25). Considering these data, *ERCC2* SNPs may serve as predictors of chemotherapy response in gastric cancer patients (26). Furthermore, two previous studies reported an association between *ERCC2* rs1799793 and survival in gastric cancer patients (17,18). However, only Li *et al* (23) reported that the rs1799793 AA genotype had a significant impact on OS in gastric cancer, which is consistent with the results of the present study.

Several limitations must be considered in the current study. Firstly, the study was conducted in a single hospital in China, and this may not sufficiently represent the entire Chinese population; selection bias may therefore have affected the results. In addition, several DNA repair pathways that may modify response to chemotherapy were analyzed; however, certain different genetic factors may influence the treatment outcome, and interaction may exist between these genes. Therefore, the results of this study require validation with larger samples. Finally, the limited sample size may also limit the statistical power to identify differences between groups. Further large sample size and multicentre studies are required to investigate the role of DNA repair genes in the clinical outcome of gastric cancer.

In conclusion, the results of the present study suggest that the *ERCC1* rs11615 and *ERCC2* rs1799793 SNPs in DNA repair pathways may be utilized as predictive factors of the clinical outcome in gastric cancer patients. In the future, these SNPs may contribute to the identification of patients who are less likely to achieve a favorable response to platinum-based chemotherapy. Translation of these pharmacogenetic predictors into clinical practice may lead to improved gastric cancer treatment planning and outcome.

## Figures and Tables

**Figure 1.** Influence of *ERCC1* rs11615 polymorphisms on overall survival of gastric cancer patients. *ERCC1*, excision repair cross-complementation group 1

**Figure 2.** Influence of *ERCC2* rs1799793 polymorphisms on survival of gastric cancer patients. *ERCC2*, excision repair cross-complementation group 2

**Table I.** Association between demographic and clinical characteristics and overall survival of gastric cancer.

Variable	Patients, n (%)	Median survival time, months	HR (95% CI)	P-value
Age, years				
<60	161 (42.37)	18.5	1.00 (ref.)	-
≥60	219 (57.63)	21.2	0.87 (0.62–1.15)	0.18
Gender				
Male	244 (64.21)	19.8	1.00 (ref.)	-
Female	136 (35.79)	20.6	0.95 (0.76–1.22)	0.16
Smoking status				
Never	214 (56.32)	23.2	1.00 (ref.)	-
Yes	166 (43.68)	15.6	1.42 (0.95–1.73)	0.11
Drinking status				
Never	172 (45.26)	22.1	1.00 (ref.)	-
Yes	208 (54.74)	16.8	1.36 (0.86–1.52)	0.08
Histological type				
Intestinal	172 (45.26)	22.5	1.00 (ref.)	-
Signet ring	164 (43.16)	20.2	1.15 (0.83–1.25)	0.25
Other	44 (11.58)	17.9	1.27 (0.72–1.39)	0.12
Histological grade				
Moderate-poor	132 (34.74)	23.4	1.00 (ref.)	-
Poor	248 (65.26)	18.6	1.22 (0.81–1.32)	0.17
TNM stage				
I–II	146 (38.42)	24.3	1.00 (ref.)	-
III–IV	234 (61.58)	15.6	2.54 (1.46–3.28)	0.007

HR, hazard ratio; CI confidence interval; ref., reference value; TNM, tumor-node-metasis (19).

**Table II.** Association between the included nine SNPs and response to chemotherapy.

	All patients		Good response (n=223)		Poor response (n=157)			
					
SNP	n	%	n	%	n	%	Adjusted OR (95% CI)	P-value
*ERCC1*rs11615								0.02
TT	173	45.53	90	40.4	83	52.87	1.00 (Ref.)	
TC+CC	207	54.47	133	59.64	74	47.13	1.66 (1.07–2.56)	
*ERCC1*rs3212986								0.05
GG	202	53.16	105	47.09	90	57.32	1.00 (Ref.)	
GT+TT	178	46.84	118	52.91	67	42.68	1.48 (0.96–2.29)	
*ERCC2*rs1799793								0.02
GG	165	43.42	86	38.57	79	50.32	1.00 (Ref.)	
GA+AA	215	56.58	137	61.43	78	49.68	1.61 (1.05–2.49)	
*ERCC2*rs13181								0.82
AA	160	42.11	92	41.26	67	42.68	1.00 (Ref.)	
AC+CC	220	57.89	131	58.74	90	57.32	1.05 (0.68–1.62)	
*NBN*rs1805794								0.39
GG	119	31.32	75	33.63	47	29.94	1.00 (Ref.)	
GC+CC	261	68.68	148	66.37	110	70.06	0.82 (0.52–1.31)	
*NBN*rs1063054								0.48
AA	171	45.00	105	47.09	68	43.31	1.00 (Ref.)	
AC+CC	209	55.00	118	52.91	89	56.69	0.86 (0.56–1.33)	
*RAD51*rs1801321								0.79
GG	135	35.53	81	36.32	55	35.03	1.00 (Ref.)	
GT+TT	245	64.47	142	63.68	102	64.97	0.94 (0.60–1.48)	
*RAD51*rs12593359								0.63
TT	147	38.68	90	40.36	59	37.58	1.00 (Ref.)	
TG+GG	233	61.32	133	59.64	98	62.42	0.90 (0.58–1.40)	
*XRCC3*rs861539								0.51
CC	242	63.68	147	65.92	98	62.42	1.00 (Ref.)	
CT+TT	138	36.32	76	34.08	59	37.58	0.87 (0.55–1.36)	

SNP, single nucleotide polymorphism; OR, odds ratio; CI, confidence interval; Ref., reference group; *ERCC1*, excision repair cross-complementation group 1; *ERCC2*, excision repair cross-complementation group 2; *NBN*, nibrin; *RAD51*, RAD51 recombinase; *XRCC3*, X-ray complementing defective repair in Chinese hamster cells 3.

**Table III.** Association between included nine SNPs and overall survival in gastric cancer patients.

			Patients, n (%)			
					
SNP	Median survival time, months	P-value (log-rank)	Survived (n=204)	Succumbed (n=176)	HR (95% CI)	Adjusted P-value
*ERCC1*rs11615						0.02
TT	23.30		82 (40.20)	91 (51.70)	1.00 (Ref.)	
TC+CC	33.20	0.017	122 (59.80)	85 (48.30)	1.71 (1.06–2.72)	
*ERCC1*rs3212986						0.04
GG	26.40		100 (49.02)	102 (50.00)	1.00 (Ref.)	
GT+TT	31.70	0.07	104 (50.98)	74 (36.27)	1.48 (0.96–2.29)	
*ERCC2*rs1799793						0.001
GG	23.10		73 (35.78)	92 (52.27)	1.00 (Ref.)	
GA+AA	34.80	0.005	131 (64.22)	84 (47.73)	1.97 (1.28–3.03)	
*ERCC2*rs13181						0.82
AA	28.90		89 (43.63)	71 (34.80)	1.00 (Ref.)	
AC+CC	29.50	0.52	115 (56.37)	105 (51.47)	1.05 (0.68–1.62)	
*NBN*rs1805794						0.39
GG	30.40		76 (37.25)	43 (21.08)	1.00 (Ref.)	
GC+CC	28.80	0.19	128 (62.75)	133 (65.20)	0.82 (0.52–1.31)	
*NBN*rs1063054						0.48
AA	31.10		104 (50.98)	67 (32.84)	1.00 (Ref.)	
AC+CC	28.90	0.13	100 (49.02)	109 (53.43)	0.86 (0.56–1.33)	
*RAD51*rs1801321						0.79
GG	32.30		85 (41.67)	50 (24.51)	1.00 (Ref.)	
GT+TT	27.60	0.21	119 (58.33)	126 (61.76)	0.94 (0.60–1.48)	
*RAD51*rs12593359						0.63
TT	30.90		91 (44.61)	56 (27.45)	1.00 (Ref.)	
TG+GG	27.10	0.25	113 (55.39)	120 (58.82)	0.90 (0.58–1.40)	
*XRCC3*rs861539						0.51
CC	30.60		138 (67.65)	104 (50.98)	1.00 (Ref.)	
CT+TT	28.30	0.43	66 (32.35)	72 (35.29)	0.87 (0.55–1.36)	

SNP, single nucleotide polymorphism; HR, hazard ratio; CI, confidence interval; Ref., reference group; *ERCC1*, excision repair cross-complementation group 1; *ERCC2*, excision repair cross-complementation group 2; *NBN*, nibrin; *RAD51*, RAD51 recombinase; *XRCC3*, X-ray complementing defective repair in Chinese hamster cells 3.
